The article "The effect of personality traits on employees’ annual salaries in Chinese startups" was retracted in 2023. Reasons: unreliable results or conclusions; concerns about the data; concerns about the results or conclusions.

# The effect of personality traits on employees’ annual salaries in Chinese startups

**DOI:** 10.3389/fpsyg.2022.1032638

**Published:** 2022-10-25

**Authors:** Longlong Zhao

**Affiliations:** ^1^School of Philosophy, Renmin University of China, Beijing, China; ^2^Department of Political Science, University College London, London, United Kingdom

**Keywords:** personality traits, annual salaries, Chinese startups, HEXACO, correlation analysis

## Abstract

Personality is a relatively regular habit of a person. It exerts a specific influence on personal behavior and the corresponding results. At the same time, personality can provide a certain degree of explanation for the differences among individuals in behavior and the related consequences. Economic differences are one of the discrepancies that exist among individuals. In order to explore the quantitative relationship between personality and individual income, this study takes 376 active employees of Chinese startups as the primary research objects. Additionally, considering the simplification and convenience of the survey, the annual salary investigated by this study is the pre-tax income of active startup employees. It uses quantitative methods to analyze the relationship between their personality traits and annual salary. Unlike the measures used in previous studies, this study employed the HEXACO-60 Inventory created by Ashton and Lee to investigate employees’ personality traits. Compared to the Big Five model, HEXACO (Honesty-Humility, Emotionality, eXtraversion, Consciousness, Open to Experience, and Agreeableness) adds a new dimension to evaluate personality traits, called Honesty-Humility (H-H). H-H did not appear in previous studies related to personality and individual income. Therefore, there is no reference to the relationship between H-H and personal earnings. Considering that the content of H-H is highly consistent with the components of inter locus of control and the core spirit advocated by the Confucian culture, which influences Chinese people profoundly, this paper proposes a bold hypothesis, that is, H-H has a positive correlation with employees’ annual salaries. Meanwhile, other corresponding hypotheses for the correlation between the other personality traits in HEXACO and employees’ annual salaries are proposed. After that, the above hypotheses are tested with the help of correlation analysis. Then, the following conclusions can be quickly drawn. Consciousness, eXtraversion, Open to Experience, and Honesty-Humility positively correlate with employees’ annual salaries. In comparison, Emotionality and Agreeableness negatively correlate with employees’ annual salaries.

## Introduction

Personality is a stable attitude of a person to reality, and the traits presented in the habitual behaviors correspond to this attitude (Nyhus and Pons, 2005). In general, personality could account for the variation of essential life outcomes of individuals (Fraley and Brent, 2005; Groves, 2005; Nyhus and Pons, 2005; Strus and Cieciuch, 2019). Relatively unfluctuating is a primary feature of personality, and it is not equal to static but a synonym of malleable (Caspi et al., 2005; Borghans et al., 2008). In other words, it is possible to make a change after an individual’s personality is formed, with the support of many indispensable prerequisites, such as enough time and efficient methods (Caspi et al., 2005; Borghans et al., 2008). Personality is a product shaped by inherited genes and objective surroundings (Nyhus and Pons, 2005). A group of experts regarded personality as an individual’s characteristics and divided it into a series of descriptive words (Denissen et al., 2018; De Haro et al., 2020). These words did make the content of personality a little bit clearer. Still, it also generated several annoying distractions in figuring out the borders and relationships of these words (Spurk and Abele, 2011). Hence some scholars recommended that a hierarchical framework could be more suitable to describe or explain what personality is (Nyhus and Pons, 2005; Spurk and Abele, 2011; Denissen et al., 2018; De Haro et al., 2020). At the same time, others argued that personality was a variational notion according to Darwin’s theory of evolution (Ng et al., 2005; Nyhus and Pons, 2005; Palifka, 2009). So, a person’s personality could be changed or molded by their surroundings (Roberts et al., 2002; Spurk and Abele, 2011; Dewaele, 2012). Although there are various definitions of personality, it is easy to make out that relative stability and conditional moldability are two apparent properties (Nyhus and Pons, 2005; Roberts et al., 2006).

In order to achieve the goal of investigating personality structure scientifically, measuring and classifying personality traits should be the first step. Asking individuals to evaluate the fitness of several targeted adjectives according to their practical situations is widely accepted as the easiest way to survey personality traits (Nyhus and Pons, 2005). Meanwhile, designing a series of behavioral questions connected with individual personality is implemental (Nyhus and Pons, 2005; Cobb-Clark and Schurer, 2012). At present, the Big Five Inventory (BFI) is the most popular method adopted by contemporary researchers (Nyhus and Pons, 2005). There are five dimensions in the BFI called “Extraversion,” “Agreeableness,” “Conscientiousness,” “Emotional Stability,” and “Autonomy” (or “Open to Experience”) (Nyhus and Pons, 2005; Cobb-Clark and Schurer, 2012). With the help of several corresponding equations, it is easy to figure out the composition of a person’s personality traits after accomplishing the BFI (Nyhus and Pons, 2005). In the late 20th century, the Big Five factors were spoken highly of by many psychological experts, and much progress was made (Nyhus and Pons, 2005; Spurk and Abele, 2011; Denissen et al., 2018). So, the BFI was regarded as a representative work for measuring personality characteristics (Nyhus and Pons, 2005; Spurk and Abele, 2011).

Nevertheless, some scholars thought that the BFI might have several potential limitations (Roberts et al., 2002; Lee and Ashton, 2004; Borghans et al., 2008; Rode et al., 2008). Thus, they kept doing lexical investigations in various languages and finally revealed that the personality variables could be cut into six factors, not just five dimensions, in the early 21st century (Ashton and Lee, 2001, 2007, 2009; Lee and Ashton, 2004). Moreover, the newly found factor differed from the traditional factors in axis location, and soon this new finding was verified and accepted by a group of researchers (Ashton and Lee, 2001; Lee and Ashton, 2004; Van Witteloostuijn et al., 2017; García et al., 2022). Although it was less popular than the Big Five, it had some merits in evaluating a person’s personality traits as a “re-organization” of BFI (Ashton and Lee, 2001, 2007, 2009; Lee and Ashton, 2004). This new discovery was called HEXACO (or the Big Six), which consisted of “Honesty-Humility” (H-H), “Emotionality” (E), “eXtraversion” (X), “Agreeableness” (A), “Conscientiousness” (C), and “Open to Experience” (O) (Ashton and Lee, 2001, 2007, 2009; Lee and Ashton, 2004).

In recent years, economists and psychologists have paid increasing attention to personality (Van Witteloostuijn et al., 2017; De Haro et al., 2020). Because they found that personality traits can be an essential indicator of predicting personal economic status, they attempted to analyze the correlation between personality traits and personal incomes (Abele and Spurk, 2009a,b; Heineck, 2011; Spurk and Abele, 2011; Denissen et al., 2018; De Haro et al., 2020). Based on their findings, research on interrelation could be cut into two different perspectives. The first research group focuses on exploring the positive/negative correlation between personality traits and personal salaries. They proved that some personality traits have a remarkable impact on individual wages and explored the attributes of this impact (Denissen et al., 2018; De Haro et al., 2020). A disagreement emerged when they were busy analyzing the exerted process and property of the mentioned influence. Some experts insisted that the firsthand impact generated by personality traits on individual earnings might be reversely negligible (Singh, 2016; Denissen et al., 2018). Based on this, they employed a moderator analysis and several mediated variables, for example, emotional intelligence, occupational self-efficacy, contractual working hours, job characteristics and so on, which could verify the influential chain of personality traits (Paunonen and Ashton, 2001; Palifka, 2009; Spurk and Abele, 2011; De Haro et al., 2020). At the same time, they revealed the indirect association between personality traits and private incomes, accompanied by many practical recommendations about how to promote personal salaries (De Haro et al., 2020). For most employees, how to boost their wages is an essential topic which draws on their immediate attention, especially for those who are hired by private companies or organizations (Spurk and Abele, 2011). In order to win a higher salary, they tried a series of approaches, such as improving their educational background, enriching personal practical experience, cultivating their specific skills and so on (Denissen et al., 2018). Although these aspects have been proven to influence the variation of their incomes, there are still lots of new indexes, for instance, personality traits, that could impact the alteration of employees’ earnings (Paunonen and Ashton, 2001; Rode et al., 2008; Denissen et al., 2018). So, some accountable recommendations for raising salaries might be distilled from how to cultivate personal personality traits.

Another research current keens on holding that the effect of personality traits on earnings is roughly ambiguous (Roberts et al., 2006; Rode et al., 2008; Palifka, 2009). Personality traits belong to a collective concept, and many constituents are included. So, it isn’t easy to declare that all personality traits significantly impact incomes (Nyhus and Pons, 2005). Duncan and Morgan (1981) approved this after they analyzed a limited number of statistics. Although a small notability influence was found between inter locus of control and earnings, a group of scholars still put the label of illegibility on their relationship (Singh, 2016; Denissen et al., 2018). In addition, if the indirect effect passed by several personality traits is considered, asserting the impact and its significance is irrational before implementing a scientific test (Borghans et al., 2008). Several scholars proved a robust association between some personality traits and productivity (Nyhus and Pons, 2005). These findings might be a supportive evidence that could verify a obvious link between several specific personality traits and earnings. However, due to the changes in datasets and metric scales, the link varies according to the concrete conditions. Therefore, it is not wise to give a general conclusion about the interrelation without considering the actual barriers created by datasets, scales and other relevant situations.

For this research, the target is to investigate the impact of personality traits on employees’ annual salaries in the range of psychological and economic literature. The economic and psychological literature have emphasized the importance of personality traits for individual incomes. Compared with the Big Five, little research adopts HEXACO as a practical tool to analyze the influence of personality traits on private annual salaries. In most relevant cases, researchers tended to investigate the effect of personality traits on salary expectation, variation of early stages’ wage, salary setting, and alteration of annual income in adult companies (Nyhus and Pons, 2005; Singh, 2016; Denissen et al., 2018; De Haro et al., 2020). Seldom did they discuss these topics in a startup scenario. Furthermore, in Chinese academia, HEXACO is not introduced (Mu et al., 2020). So, it is impossible to find a Chinese scholar who dissects the personality structure of Chinese people with the help of HEXACO. From these perspectives, this article might be comparatively innovative and creative.

This research intends to analyze the personality structure of employees in Chinese startups first and then assess its impact on individual annual salary directly. Under the direction of these psychological methods, it is easy to find the “successful personality traits” that share a significant association with economic achievement. More specifically, the more remarkable a person’s “successful personality traits,” the more likely he/she is to get a higher wage monthly or annually. Thus, it is cushy to draw a personality portrait of the ideal employees after elemental analysis statistically. That way, it provides more convenience for job seekers and employers to promote their careers and profit from the personality perspective.

According to the results of this research, it is easy to draw the following conclusion in Chinese startups. Honesty-Humility, eXtraversion, Consciousness, and Open to Experience have a positive correlation with employees’ annual salaries, while Emotionality and Agreeableness has a negative correlation with employees’ annual salaries.

The remainder of this study will be developed in the following order: Section “Literature review” reviews the central literature connected with personality traits and personal income, and advocates six main assumptions about the correlations of personality traits (measured by HEXACO) and personal income. Section “Data and methodology” lists the primary methodology used by this research and offers a general description of how to conduct the survey. Section “Findings” displays the key findings. Section “Conclusion” concludes the conclusions. In addition, the original questionnaires are provided in Appendices 1, 2.

## Literature review

The premise of promoting current research is to master the primary situation of the existing findings in a related field (Mu et al., 2020). Therefore, to sort out the results focusing on “the influence of personality traits on employees’ annual salaries in Chinese startups” more comprehensively, this section will be further refined into three parts. The first part mainly concerns the mainstream called “measurable scales of personality traits.” It introduces the content of the Big Five and HEXACO, which are currently widely used and relatively influential scales. Meanwhile, some important comparisons of them also have been made in this part. The second part focuses on the interrelationship between personality traits and individual salary, and highlights several types of viewpoints connected with the relationship. Then, six hypotheses related to six personality traits (HEXACO) and employees’ annual salaries (before tax) in Chinese startups have been put forward. The third part concentrates on introducing the social context of Chinese startups, and the reasons why this study chose it as a primary scenario.

### Metrical scales of personality traits

In the early days, Personality was a research topic in linguistics (Ashton et al., 2004b; Saucier, 2009; Strus and Cieciuch, 2019). As an important distinction between people, personality traits were used by lexicologists through different adjectives to mark different people (Allport and Odbert, 1936; Thalmayer et al., 2019). In order to accurately describe personality traits, linguists found thousands of adjectives in lexical dictionaries (Ashton et al., 2004a). Due to its excellent content, the descriptive corpus of human personality traits brought much inconvenience to theoretical research and practical operation (Thalmayer et al., 2019). Thus, some researchers began to investigate how to compress the corpus (Saucier, 2009). The personal personality traits test scale is a significant research result obtained by these researchers (Allport and Odbert, 1936; Thalmayer et al., 2019). Through the unremitting efforts of researchers, more and more personality scales had been created and applied to practice, such as the BFI and the HEXACO Inventory, which have been accepted in a broader range. From the perspective of acceptance and application, the BFI was undoubtedly second to none not so long ago. And the HEXACO Inventory is a relatively new scale with certain developmental potential, because it contains several innovative features which could make it advantageous compared with the Big Five (Ashton et al., 2004b; Saucier, 2009).

#### Big Five model

Allport and Odbert (1936) proposed a famous lexical hypothesis. They argued that the most important differences between individuals could be described by those adjectives that characterize personality traits. As a result, they further reduced these adjectives describing personality traits from 17,953 to 4,504, laying a solid foundation for forming the Big Five personality traits (Allport and Odbert, 1936). Then other linguists and psychologists began to copy them (Allport and Odbert, 1936). After a period of development, those adjectives that describe personality traits were gradually summarized as five superordinate factors (Ashton et al., 2004a; Saucier, 2009). The man who made these five dimensions the famous Big Five was Goldberg (1971). Goldberg (1971) officially named the five factors that characterize personality traits as “OCEAN”. Specifically, “OCEAN” refers to Open to Experience (or Intellect/Culture), Conscientiousness, Extraversion, Agreeableness, and Neuroticism (or Emotional Stability). Each of the above five dimensions contains several characters that could describe a specific aspect of personality traits. Subsequently, the ability of “OCEAN” to assess individual personality traits had been repeatedly tested and generally recognized by many researchers, such as John, Costa, McCrae, Srivastava, and so on (Costa and McCrae, 1988; McCrae and Costa, 1994, 1996; John and Srivastava, 1999). They believe there is a degree of mapping relationship or correlativity among the five dimensions (McCrae and Costa, 1996; John and Srivastava, 1999). It is worth mentioning that Costa and McCrae revised the inventory of the Big Five in 1992, resulting in a version containing five main dimensions, each of which contained six facets (Costa and McCrae, 1992b). After this revised version came out, it was not only favored by most scholars but also became the most widely used and most popular Big Five questionnaire in history (Costa and McCrae, 1992a,b; Judge et al., 1999; Ludeke et al., 2019). At the same time, in naming the five dimensions, experts represented by Digman (1990), Barrick and Mount (1991), and Salgado (1997) disagreed with scholars represented by Costa and McCrae (1992a), John and Srivastava (1999), etc., especially in defining the first dimension. The former thinks it should be labeled “Autonomy,” but the latter insists on labeling it “Open to Experience.” Although both views have some supporters, in fact the latter have a significant advantage in terms of application and popularity.

The Big Five is not a flawless masterpiece. There are plenty of criticisms surrounding its shortcomings. According to the content of these criticisms, they can be roughly divided into the following categories: Firstly, theoretical criticisms. Some scholars believed that there may be more than five personality traits in reality for a person (Mershon and Gorsuch, 1988). At the same time, a person’s personality traits may also be summarized by two or three factors (Tellegen, 1985; Cloninger, 1987; Digman, 1990; Eysenck, 1991). In addition, the Big Five had been criticized for its lack of measures of motivation (Ashton and Lee, 2007). Lately, with the continuous improvement of research, Roberts et al. (2006) gave a relatively comprehensive explanation of the differences in metrical methods and research strategies between motivation and personality traits. So the critique of the Big Five from the motivation perspective gradually mediated. Secondly, atheoretical criticisms. They were the harshest type of criticism the Big Five had faced. They sharply pointed out an essential flaw in the Big Five, that is, it lacks of support from fundamental theories. Considering all the questions in the Big Five scale, the responses that a person would make are based on a hypothetical situation (Nyhus and Pons, 2005; Ashton and Lee, 2007; Borghans et al., 2008; Denissen et al., 2018). So, these questions lack the necessary realistic basis (Borghans et al., 2008; Denissen et al., 2018). Therefore, a particular deviation between the test results and the on-the-spot reaction of a person in the actual situation could be created (Nyhus and Pons, 2005; Ashton and Lee, 2007).

The wide variety of personality tests and the lack of consensus were two major problems faced by the Big Five in practical application (Nyhus and Pons, 2005; Ashton and Lee, 2007; Borghans et al., 2008; Denissen et al., 2018). Additionally, Block (1995) not only questioned the Big Five scale but also questioned the practice of using factor analysis to explore the structure of personality. He believed that the scale involves some personal items, so the objectivity of the results would be disturbed or challenged to varying degrees (Block, 1995). Different scholars had different views on each factor in the Big Five. For example, on attributing impassivity, Costa and McCrae (1992b) declared that it was a part of Neuroticism. However, Revelle (1997) argued that it was a mixture of Neuroticism, Consciousness and Neuroticism. Despite some drawbacks to the Big Five, many scholars still would like to use it to estimate personality traits in practice (Little et al., 1992; Judge et al., 1999; Ludeke et al., 2019).

#### HEXACO

The Big Five was further expanded with the continuous deepening of the lexical research on personality structure (Ashton, 1998; Lee and Ashton, 2004; Ashton and Lee, 2007; Ashton et al., 2014). In the early 21st century, Ashton and Lee proposed a six-dimensional model for measuring personality traits based on summarizing a large amount of real-world evidence, namely HEXACO (Ashton and Lee, 2001, 2007; Lee and Ashton, 2004; Ashton et al., 2014). HEXACO is mainly composed of six factors, and they are Honesty-Humility (H-H), Emotionality (E), eXtraversion (X), Agreeableness (A), Consciousness (C), Open to Experience (O) (Ashton and Lee, 2009). Table 1 is a brief introduction and interpretation of the main content of HEXACO, and for more specific details, see the article written by Lee and Ashton (2004).

**TABLE 1:** The main facets and interpretations of the HEXACO Inventory.

Factors	Facets	High score	Low score
Honesty-Humility	Sincere	Unwilling to manipulate others	Flatter others to gain favors
	Fairness	Unwilling to utilize others at large	Willing to gain by fraud/corruption
	Greed avoidance	Not especially motivated by monetary/social-status	Tend to enjoy/display wealth/privilege
	Modesty	View themselves as the general public	Consider themselves as unusual privileges
Emotionality	Fearfulness	Avoid physical harm strongly	Fearlessness toward physical harm
	Anxiety	Be preoccupied toward minor problems	Feel little stress toward difficulties
	Dependence	Share their difficulties with friends	Self-confident and independence
	Sentimentality	Strong emotional attachments and empathy	Little emotion and unconcern others
eXtraversion	Expressiveness	Dramatic (speaking) and talkative	Behave poorly in oral expression
	Social boldness	More boldness in social occasions	Feel shy and awkward in public
	Sociability	Enjoy talking, visiting and social activities	Prefer solitary activities and less conversation
	Liveliness	Optimism and high spirit	Less cheerful/dynamic
Agreeableness	Forgiveness	Forgive offenders and re-build relations	Hold a grudge toward offenders
	Gentleness	Judge others gently	Evaluate others critically
	Flexibility	Avoid arguments and tolerate different views	Tend to be argumentative and stubborn
	Patience	Tend to be more patient	Easy to lose their tempers
Consciousness	Organization	Tend to be tidy/structured	Tend to be sloppy/haphazard
	Diligence	More diligent	Little self-discipline
	Perfectionism	Chase for perfectionism	Tolerate some errors
	Prudence	Be cautious and self-controlled	Act impulsively
Open to Experience	Aesthetic appreciation	Strong enjoyment of beauty	Less enjoyment of beauty
	Inquisitiveness	Be interested in travel and read widely	Little curiosity about the natural/social sciences
	Creativity	Be filled with creativity	Lack of original though
	Unconventionality	Accept seemingly strange/radical ideas	Avoid eccentric/non-conforming persons

These contents come from HEXACO-Personality Inventory-Revised (Lee and Ashton, 2004; Ashton and Lee, 2009).

Compared to the Big Five, HEXACO is more responsive in different cultural environments (Lee and Ashton, 2008, 2012, 2013; Saucier, 2009). And HEXACO struggled to respond well in all cultural contexts (Skimina et al., 2020). From the available findings, only Social Self-Regulation (Conscientiousness, Honesty-Humility, and Agreeableness) and Dynamism (Openness to Experience and eXtraversion) can be free from the shackles of the cultural context in the process of application (Saucier et al., 2014; Saucier and Srivastava, 2015; Strus and Cieciuch, 2019; Thalmayer et al., 2019). As for Emotionality, it was more complicated and could be found in Dynamism or from Social Self-Regulation (De Raad, 2009; Saucier, 2009; De Raad et al., 2010; Saucier et al., 2014; Saucier and Srivastava, 2015). In addition, another advantage of HEXACO over the Big Five is that it includes some variables that have not yet been covered by the Big Five, such as Honey-Humility (H-H) (Lee and Ashton, 2012, 2013, 2018; Ashton et al., 2019; Ludeke et al., 2019). H-H is not the only factor in HEXACO that differentiates from the Big Five (Lee and Ashton, 2012, 2013, 2018; Ashton et al., 2019). Specifically, Agreeableness and Emotionality in HEXACO are rotational variants of Neuroticism and Agreeableness in the Big Five, respectively (De Vries et al., 2008). Agreeableness and Emotionality in HEXACO are more extensive than those in Neuroticism and Agreeableness in the Big Five (Lee and Ashton, 2005; Ashton and Lee, 2007; De Vries et al., 2009; Hilbig et al., 2013; Hilbig and Zettler, 2015; Skimina et al., 2018). While the remaining factors in HEXACO are not distinct from those corresponding dimensions in the Big Five (Ashton and Lee, 2007).

HEXACO Personality Inventory-Revised is a popular metrical method currently, and it can be divided into three versions, called 200-version, 100-version, and 60-version, according to the number of questions in the questionnaire (Lee and Ashton, 2004, 2012, 2013, 2018; Ashton and Lee, 2009). In particular, the 100-version and 60-version are the most frequently used scaled in personality traits studies and are favored by many researchers (Lee and Ashton, 2018). As for this study, the 60-version is employed to investigate the personality traits of employees in Chinese startups.

### The association between personality traits and individual income

Previous empirical studies focused on analyzing the causes of wage differentials between workers from the perspective of human capital, job training, or formal demography (Filer, 1981; Goldsmith et al., 1997; Palifka, 2009; Denissen et al., 2018). While these perspectives have been shown to help explain wage differentials, many other factors that contribute to wage differentials need to be explored (Palifka, 2009; Denissen et al., 2018). In order to fully understand the causes of wage differences between workers, some economists began to investigate the impact of personality traits on wages (Ferris et al., 2001; Dilchert and Ones, 2008; Denissen et al., 2018). In general, researchers tended to mainly use the Rotten scale, the Big Five, or other scales to investigate employees’ personality traits (the HEXACO scale has not yet been found to be used in these studies currently), and then they focused on analyzing the correlation between personality traits and personal income (Dilchert and Ones, 2008; Denissen et al., 2018).

Judging from the current research results, the discussion of the relationship between personality traits and personal income revolves around the correlation between specific facets of personality traits and individual income, or the influence of the former on the latter (Ferris et al., 2001; Dilchert and Ones, 2008; Denissen et al., 2018). At the end of the 20th century, scholars demonstrated the conclusion that psychological capital, which contains internal locus of control and personality traits, exerts an extraordinary and vital impact on personal income (Jencks, 1979; Duncan and Morgan, 1981; Goldsmith et al., 1997; Bowles et al., 2001a,b). At the same time, research on the relationship between certain specific personality traits and personal incomes had been developed accordingly (Dilchert and Ones, 2008; Denissen et al., 2018). For example, Filer (1981) discovered that four personality traits uniquely affect individual salary. Goldsmith et al. (1997) found that changes in self-esteem were more likely to cause changes in an individual’s income than changes in human capital. Duncan and Dunifon (1998) divided personality traits into motivational and behavioral traits, proving that both significantly impacted personal income. Osborne (2000) pointed out that the impact of personality traits on individual income could also be significantly different due to the difference between gender and automotive status. After operating empirical research, Nyhus and Pons (2005) discovered that there was a series of significant correlations between the three factors in the Big Five (namely, Emotional Stability, Agreeableness, Conscientiousness) and employees’ wages, and these correlations had significant gender differences.

After looking at all the quantitative studies regarding the Big Five as the primary measurement tool, it is easy to see that researchers had a significant disagreement when discussing the impact of personality traits on personal wages (Dilchert and Ones, 2008; Denissen et al., 2018). Some researchers believed that in addition to Openness to Experience, the other four personality traits have a significant positive/negative effect on employees’ wages (Judge et al., 1999; Ferris et al., 2001; Waldman and Korbar, 2004; Ng et al., 2005; Nyhus and Pons, 2005; Gelissen and de Graaf, 2006; Dilchert and Ones, 2008; Rode et al., 2008; Palifka, 2009; Sutin et al., 2009). Others argued that the impact of personality traits on personal wages was indirect (Hogan, 1983; Cantor, 1990; Little et al., 1992; Lent et al., 1994; McCrae and Costa, 1996; Boudreau et al., 2001; Zhang and Arvey, 2009; Spurk and Abele, 2011). In conclusion, Agreeableness, Conscientiousness, Emotional Stability, Autonomy, Extraversion, Neuroticism, and Openness to Experience have all been shown to have a positive/negative correlation with individual income. For the specific correlation between the above personality traits and individual incomes, please see Table 2.

**TABLE 2:** Correlations between personality traits in the Big Five and the annual income.

Personality traits	Effect on (association with) earnings
**Agreeableness**	Positive (Turner and Martinez, 1977) Negative (Judge et al., 1999; Ferris et al., 2001; Waldman and Korbar, 2004; Ng et al., 2005; Nyhus and Pons, 2005; Gelissen and de Graaf, 2006; Hülsheger et al., 2006; Dilchert and Ones, 2008; Rode et al., 2008; Palifka, 2009; Sutin et al., 2009)
**Conscientiousness**	Positive (Barrick and Mount, 1991; Salgado, 1997; Judge et al., 1999; Ferris et al., 2001; Waldman and Korbar, 2004; Ng et al., 2005; Nyhus and Pons, 2005; Gelissen and de Graaf, 2006; Hülsheger et al., 2006; Dilchert and Ones, 2008; Rode et al., 2008; Palifka, 2009; Sutin et al., 2009)
**Emotional stability**	Positive (Barrick and Mount, 1991; Salgado, 1997; Judge et al., 1999; Ferris et al., 2001; Waldman and Korbar, 2004; Ng et al., 2005; Nyhus and Pons, 2005; Gelissen and de Graaf, 2006; Hülsheger et al., 2006; Dilchert and Ones, 2008; Rode et al., 2008; Palifka, 2009; Sutin et al., 2009)
**Autonomy**	Positive (Filer, 1981; Nyhus and Pons, 2005)
**Extraversion**	Positive (Judge et al., 1999; Ferris et al., 2001; Waldman and Korbar, 2004; Ng et al., 2005; Nyhus and Pons, 2005; Gelissen and de Graaf, 2006; Hülsheger et al., 2006; Dilchert and Ones, 2008; Rode et al., 2008; Palifka, 2009; Sutin et al., 2009)
**Neuroticism(^©^**	Negative (Judge et al., 1999; Ferris et al., 2001; Waldman and Korbar, 2004; Ng et al., 2005; Nyhus and Pons, 2005; Gelissen and de Graaf, 2006; Hülsheger et al., 2006; Dilchert and Ones, 2008; Rode et al., 2008; Palifka, 2009; Sutin et al., 2009)
**Openness to experience**	Positive (Judge et al., 1999; Ng et al., 2005) Not found (Barrick and Mount, 1991; Salgado, 1997; Ferris et al., 2001; Waldman and Korbar, 2004; Nyhus and Pons, 2005; Gelissen and de Graaf, 2006; Hülsheger et al., 2006; Dilchert and Ones, 2008; Rode et al., 2008; Palifka, 2009; Sutin et al., 2009)

Indicates that this facet could be found in some scales sometime. A scale usual contains autonomy, it would exclude open to experience.

(^©^Indicates that this facet could be replaced by emotional stability in some scales sometime.

From the available research results, most researchers agreed that Conscientiousness, Extraversion, and Emotional stability all generated positive impacts on individual earnings (shown in Table 2). However, when discussing the correlation or interaction between Agreeableness and personal income, scholars clearly disagreed. Most researchers have demonstrated empirical analysis that Agreeableness negatively impacted personal income. In contrast, only a smaller group of researchers insisted that the effect was negative. A similar situation happens when talking about the connection between Open to experience and individual salaries. Some researchers claimed that no link had been found. However, another group of researchers found a conclusion after analyzing the survey. They claimed that Open to experience had a positive impact on individual salaries. As for the extent to which H-H affects earnings, no researcher has yet given an empirical argument. Most previous studies that discussed the relationship between personality and income were focused on using the Big Five, so they measured five main personality traits. H-H is different from any of the personality traits in the Big Five. Therefore, it is difficult to find empirical studies that specifically explore the quantitative relationship between H-H and personal annual income. In order to make a relatively reasonable assumption about this quantitative relationship, the author collected the behavior habits of the targeted respondents in dealing with problems on a daily basis during the offline interviews. “Integrity, cooperation, sense of responsibility, and personal cultivation” were the four expressions that the interviewees used to describe their daily habits or basis for processing usual things. Combined with Chinese cultural traditions, it can be seen that Confucian culture exerts a deep-rooted influence on the daily life and behavioral customs of Chinese people (Zhang et al., 2003; Xiu et al., 2015). Confucian culture advocates improving personal cultivation, adhering to honesty and trustworthiness, strengthening teamwork, and taking on social responsibilities (Zhang et al., 2003; Xiu et al., 2015). It can be seen that the content advocated by Confucian culture coincides with some components of H-H. After considering the relationship between other personality traits with altruistic attributes and personal income, the influence delivered by H-H could be figured out probably. In addition, according to the description of H-H shown in Table 1, some parts of it could be included by the internal locus of control (Ludeke et al., 2019; Strus and Cieciuch, 2019). Therefore, the effect of H-H on earnings might be roughly inferred from the correlation between the internal locus of control and earnings (De Haro et al., 2020; Kräft and Urgelles, 2021; García et al., 2022). Some researchers believed that internal locus of control positively affected earnings (De Haro et al., 2020; Kräft and Urgelles, 2021; García et al., 2022), while several argued that this effect was negative (Kräft and Urgelles, 2021; García et al., 2022). Furthermore, limited researchers reckoned that the correlation between them was ambiguous (Denissen et al., 2018). All in all, based on the above analysis and the description of HEXACO in Table 1, six hypotheses could describe the relationship between personality traits in HEXACO and personal income in Chinese startups. They are as follows:

Hypothesis 1: Consciousness has a positive correlation with employees’ annual salaries.

Hypothesis 2: eXtraversion has a positive correlation with employees’ annual salaries.

Hypothesis 3: Emotionality has a negative correlation with employees’ annual salaries.

Hypothesis 4: Agreeableness has a negative correlation with employees’ annual salaries.

Hypothesis 5: Open to Experience has a positive correlation with employees’ annual salaries.

Hypothesis 6: Honesty-Humility has a positive correlation with employees’ annual salaries.

### The social context of Chinese startups and reasons for setting

Starting a new company is challenging and relies on a prominent team (Chen, 2004; Hu and Zhou, 2011). A benign social environment and the joint efforts of team members are two critical factors for a startup to survive (refers to making profits continuously) (Le et al., 2012; Li et al., 2012). Most Chinese startups have been in a benign social environment since 2018 (Chen et al., 2021; Zhang et al., 2021). Precisely, this favorable social environment consists of three aspects. Firstly, more robust support is given by the government. Since 2018, the Chinese government has successively issued numerous “guidance opinions” and “preferential policies” to encourage citizens to start their businesses (Yang et al., 2014; Zhong, 2015). The support for startups in taxation and finance has been increasing yearly (Wang, 2016; Zhong et al., 2016). Secondly, the enthusiasm of Chinese citizens to start a business is rising gradually, and the number of entrepreneurs is growing annually (Ji and Liu, 2016; Zeng and Li, 2017; Chen et al., 2021). The proportion of entrepreneurs with bachelor’s degrees or above is also climbing (Chen et al., 2012, 2021; Liu and Tang, 2014; Zhang et al., 2021). Thirdly, the social recognition of entrepreneurs is improving persistently. The public generally has a recognized and approved attitude toward entrepreneurs and joining a startup (Tang, 2021; Yin, 2021). In short, the current entrepreneurial environment in China is relatively favorable on the whole. Therefore, choosing startups as the research point is more in line with the trend of contemporary development in China. After that, studies have shown that startups can quickly recruit a group of employees with certain character traits or ethos (Li, 2012; Wang et al., 2022). For example, startups could attract passionate, creative and innovative candidates (Lei et al., 2011; Li, 2011; Wang et al., 2022). Fourthly, some Chinese scholars linked the success of startups and their employees’ personality traits and believed there might be a close relationship between the two (Guo, 2011; Qi and Liu, 2011; Wang et al., 2022). Therefore, selecting Chinese startups as a trigger could promote the process of further exploring the above relationship. In addition, most of the relevant research tends to pick up mature companies or general corporations as their research points (Hu and Zhou, 2011; Zeng and Li, 2017; Yin, 2021), seldom do they pay attention to startups. Therefore, this research concentrate on Chinese startups, which could expand the scope of current research at the level of startups.

## Data and methodology

In order to accurately investigate the influence of personality traits on individual wages, it is important to know that some variables, such as the job position, and education level, may influence personal salary. As for other factors that could have an impact on personal income, such as personal appearance (Kräft and Urgelles, 2021; García et al., 2022), height (Kräft and Urgelles, 2021; García et al., 2022), weight (Kräft and Urgelles, 2021; García et al., 2022), family background (Ludeke et al., 2019; Kräft and Urgelles, 2021; García et al., 2022), working experience (Strus and Cieciuch, 2019; García et al., 2022), religious beliefs (Kräft and Urgelles, 2021; García et al., 2022), due to their absence in current survey, this study “suppose” that they were no apparent differences in these aspects. The so-called “suppose” is a basic assumption and an essential premise for this research to maintain a high degree of scientificity and rationality. Because many scholars have verified the influence of the above factors on individual wages, it is necessary to make a certain degree of limitation and explanation before implementing data analysis commands (Strus and Cieciuch, 2019; Kräft and Urgelles, 2021).

### Data and sources

The six hypotheses proposed in this paper can be tested only when the appropriate amount of data is collected. So, after completing the design of the questionnaire (see Appendices 1, 2), the author emailed more than 380 employees of 56 startups in China. The startups in China studied in this survey mainly refer to those established between January 1 and December 31, 2018, and have been profitable from their establishment until May 31, 2022. Usually, these enterprises’ employees are less than 100, and their business scope mainly concentrates on Internet technology, educational training, and talent agent. Overall, the online survey took about a month and a half. It distributed 386 questionnaires and recovered 380, of which 376 were valid. This high response rate is mainly due to the fact that the author actively visited the targeted startups and had a communication with every participants. The online questionnaire evaluate the personality traits of employees in Chinese startups. At present, in the fields of psychology, economics and management, it is rare to find research related to exploring the impacts of personality characteristics of employees in Chinese startups on their economic incomes with the help of the HEXACO-60 scale. Compared with the application range and frequency of the Big Five scale, the HEXACO scale still has much potential for popularization and application. In China, the research around HEXACO is in its infancy (Mu et al., 2020). Therefore, this study promotes the scope of HEXACO to a certain extent and makes a few contributions to promoting HEXACO in China.

Using a personality scale to investigate the personality traits of a specific research subject (such as undergraduates, graduates, employees, etc.) has become a significant option made by relevant researchers (Ludeke et al., 2019; Strus and Cieciuch, 2019; Kräft and Urgelles, 2021; García et al., 2022). However, it does not mean that their choices do not have any drawbacks in practice. For example, due to the influence generated by the method and content of a survey, or the other factors (such as social scene, cultural traditions, and so on), there would inevitably be a difference between the personality characteristics reflected finally by the questionnaires and the essential personality traits of a specific object (Ludeke et al., 2019; Kräft and Urgelles, 2021; García et al., 2022). Indeed, this difference could be gradually narrowed with research methods and relevant technology optimization (Strus and Cieciuch, 2019; García et al., 2022). At the same time, one of the most significant advantages of adopting this approach is that an analysis of the personality characteristics of particular objects can be achieved quickly (Ludeke et al., 2019; García et al., 2022). This article uses HEXACO-60 to conduct a more detailed survey of employees’ personality traits and their annual incomes. When investigating employees’ annual income, the authors selected their pre-tax income. This is because it can improve the investigation’s convenience and efficiency while avoiding the troubles caused by tax calculations or other issues. More than 370 active employees of Chinese startups took part in the offline interviews. The offline interviews measured five aspects in detail, namely the gender, year of birth, education level, position, annual salary. Compared with similar investigations in the past, the personality scale selected in this survey is more informative, and the respondents are more targeted. This study did not contain factors such as the respondents’ stature, appearance, family background, etc. Some researchers have shown that these factors could affect an employee’s income significantly (Ludeke et al., 2019; Strus and Cieciuch, 2019; Kräft and Urgelles, 2021; García et al., 2022). Therefore, from this point of view, there are certain shortcomings in this study. Compared with those without working experience, the personality of active employees is more likely to be affected by working scenarios, relationships, and organizational culture (Ludeke et al., 2019; Strus and Cieciuch, 2019). Moreover, regarding personal ability, personality characteristics, work style, etc., active employees of entrepreneurial companies are more recognizable than employees of non-entrepreneurial companies in general (Ludeke et al., 2019; Strus and Cieciuch, 2019; Kräft and Urgelles, 2021; García et al., 2022). Thus, considering the particularities of active employees in Chinese startups, the advantages of conducting personality surveys of active employees and the innovation, the advantages of this survey are far more significant than their disadvantages.

When using questionnaires to collect the independent and dependent variables needed for the study from the same respondents, common method variance (CMV) was easy to emerge (Van Witteloostuijn et al., 2017). Because the measurement tools used were the same. Although the CMV does not necessarily bias the results, as the degree of similarity of measurement methods increases, it is more likely to induce bias in the results (Van Witteloostuijn et al., 2017). If the same measurement tool or method is used to raise the data required, the probability of deviation in the final research results would be increased (Van Witteloostuijn et al., 2017). Therefore, when analyzing the relationship between independent and dependent variables, minimizing the potential adverse effects caused by the CMV is necessary (Van Witteloostuijn et al., 2017).

In order to effectively avoid the risk of CMV, weakening the singularity of data sources and the similarity of measurement methods is a practical strategy for general researchers (Van Witteloostuijn et al., 2017). Therefore, two different types of questionnaires were employed when collecting the data needed for this article. The first type of questionnaire was designed to investigate the personality traits of active employees, and the second one was created to survey the basic information of active employees (including their annual salary before tax). In early June 2022, the author emailed more than 380 active employees the first online questionnaire, in order to explore their personality traits. By the end of June, 380 responses were received. Three weeks later, with the assistance of a group of HR managers, the author distributed paper questionnaires to the same group of active employees who had filled out the online questionnaires and surveyed their gender, year of birth, education level, position, and annual salaries. With the help of two different methods, the statistics of relevant variables (such as, employees’ personality traits, employees’ annual incomes before tax, etc.) were collected. Thus, the need to minimize the “biased” effects of the CMV as much as possible could be fulfilled. In addition, all the online surveys and offline questionnaires in this study were conducted ethically.

### Measures

In general, an employee’s gender, age, level of education, position, family background, and appearance could affect their financial situation to varying degrees (Borghans et al., 2008; Denissen et al., 2018; De Haro et al., 2020). If all these factors are included in the statistical scope of the questionnaire, it will undoubtedly have a positive impact on improving the comprehensiveness and scientific nature of the research. However, at the same time, it will also bring many difficulties and inconveniences to data collection and analysis. In most empirical studies, researchers preferred to choose a limited number of factors as the leading indicators to investigate (Denissen et al., 2018; De Haro et al., 2020). Therefore, this study selected the gender, age, education level, position and personality traits of employees as key indicators. As for other indicators, such as family background, appearance, etc., these are not taken into account for the time being. Indeed, this choice may cause some degree of interference to the accurate output of the final results. Therefore, when selecting the targeted employees, the author tried to artificially exclude those with significant differences in appearance and family background as much as possible. Although the influence generated by the other factors cannot be wholly excluded in this way, it weakens the resulting interference to a certain extent, at least.

The survey consisted of two main sections. The first section is to send online questionnaires to employees of startups in the form of e-mails to investigate their personality traits. The online questionnaires were dominated by the HEXACO-60 Inventory created by Ashton and Lee (2009). Please refer to Appendix 2 for a detailed personality questionnaire. Specifically, the online questionnaire mainly contains six personality traits, each of which corresponds to 10 questions, and each question uses a Likert Type of Scale, and the corresponding value increases from 1 (representing “strongly disagree”) to 5 (representing “strongly agree”). In addition, questions 1–10 measure H-H, questions 11–20 measure E, questions 21–30 measure X, questions 31–40 measure A, questions 41–50 measure C, and questions 51–60 mainly measure O. After collecting all data related to personality traits, the authors tested the Cronbach’s α with the help of Stata, a comprehensive statistical software, and found the Cronbach’s α of Honesty-Humility, Emotionality, eXtraversion, Agreeableness, Consciousness, and Open to Experience are 0.83, 0.85, 0.87, 0.82, 0.84, and 0.86. Thus, the database related to personality traits has a high credibility.

The second section is to conduct offline interviews with all active employees who have received online questionnaires to collect statistics on their gender, year of birth, level of education, position and annual income (before tax). The offline interview questionnaire contains five dimensions. For details, please refer to Appendix 1. The first dimension of it is the gender of the employee. For this dimension, number 1 represents male, and number 2 represents female. The second dimension is the employee’s age, which mainly counts the employee’s birth year. This question is a fill-in-the-blank question; the employee fills in the specific birth year according to their actual situation. After counting the collected data for this question, it is easy to divide them into three ranges, namely numbers 1 (18–24 years old), 2 (25–30 years old), and 3 (31–40 years old). The third dimension is the employees’ level of education, and the numbers 1, 2, 3, 4, and 5 represent Undergraduate students, Bachelors, Master students, Masters, PhD students/Doctors. The fourth dimension is the position of an employee, and the numbers 1, 2, 3, 4, and 5 represent a general clerk (the ground level of a company), a supervisor (mainly responsible for managing general clerks), a manager (mainly responsible for leading the supervisors), a Director (mainly responsible for directing managers), a copartner (refers to the partner of the company) respectively. The fifth dimension is the employee’s annual income (before tax) distinguished by number 1 (Less than 12,000 British pounds), 2 (12,001–24,000 British pounds), 3 (24,001–36,000 British pounds), 4 (36,001–48,000 British pounds), and 5 (Over 48,001 British pounds). After collecting all the relevant data for the above dimensions, the authors tested the Cronbach’s α of the dataset with the help of Stata and found that the Cronbach’s α of the offline interview questionnaire was 0.81. So, this dataset has a high degree of reliability.

In addition, Table 3 is a statistical description of all the variables. According to the presented standard deviations and means in this table, the standard deviation of Q1 is the same as Q2, but their corresponding means are different (the mean of Q2 is larger). At the same time, H-H, E, X, A, C, and O have the same standard deviation, but their means are not entirely consistent. Specifically, H-H, X, C, and O share a mean, and so do E and A.

**TABLE 3:** Statistical description of main variables.

Variable	Mean	Standard deviation	Minimum	Maximum
Biological gender	1.470	0.500	1	2
Age	1.890	0.500	1	3
Education level	2.200	1.270	1	5
Position	2.410	1.340	1	5
Annual salary	2.200	1.070	1	5
H-H	3.790	0.280	3.500	4.500
E	2.210	0.280	1.500	2.500
X	3.790	0.280	3.500	4.500
A	2.210	0.280	1.500	2.500
C	3.790	0.280	3.500	4.500
O	3.790	0.280	3.500	4.500

## Findings

According to the final statistical results of the offline interview, a total of 376 employees from different startups participated in China. First of all, from the perspective of gender composition, there were 198 male participants, accounting for 52.66%. Moreover, there were 178 female participants, accounting for 47.34%. It can be seen that the gender ratio of respondents is in a state of elemental balance. Secondly, from the perspective of the education level, college students (accounting for 34.04%) and bachelors (42.55%) are the main force of the investigated Chinese startups. In contrast, fewer than 16 and 0.1% of master’s and PhD/PhD students were surveyed. Then, in terms of the age of the participants, nearly 73.67% were between 25 and 30 years old, 18.62% were between 18 and 24, and about 7.71% were between 31 and 40. It is worth noting that among all those involved in the survey, no participant is older than 40. Next, from the view of participants’ positions, 128 general clerks, 90 supervisors, 70 managers, 50 directors, and 38 copartners participated in the survey. From these statistics, it is easy to see that employees of the vast majority of positions participated in the survey. Finally, in terms of the annual income (before tax), there were 128 employees in the “first class” (Less than 12,000 pounds), 90 employees in the “second class” (12,001–24,000 pounds), 120 employees in the “third class” (24,001–36,000 pounds), 29 employees in the “fourth class” (36,001–48,000 pounds), and nine employees in the “fifth class” (Over 48,001 pounds).

Figures 1–6 show a visible positive correlation between H-H and annual salary regarding their variation trends, and a similar correlation exists between X and annual salary, between C and annual salary, and between O and annual salary. However, there is a visible negative correlation between E and annual salary and a semblable correlation between A and annual salary. Based on these, it can be inferred that if there is a growth momentum in annual salary, then H-H, X, C, and O are likely to show a corresponding trend of being strengthened, and E and A may show a related trend of being weakened.

**FIGURE 1:** Annual salary and H-H.

**FIGURE 2:** Annual salary and E.

**FIGURE 3:** Annual salary and X.

**FIGURE 4:** Annual salary and A.

**FIGURE 5:** Annual salary and C.

**FIGURE 6:** Annual salary and O.

From Figures 7–12, it can be seen that there is a positive visual correlation between H-H and job position, and a similar correlation exists between X and job position, between C and job position, and between O and job position. In contrast, there is a visual negative correlation between E and job position and a semblable correlation between A and job position. Based on these, it can be inferred that if the job position has a current of growth (refers to the promotion of the job position), then H-H, X, C, and O are likely to show a corresponding trend of being strengthened, and E and A may show a related trend of being weakened.

**FIGURE 7:** Job position and H-H.

**FIGURE 8:** Job position and E.

**FIGURE 9:** Job position and X.

**FIGURE 10:** Job position and A.

**FIGURE 11:** Job position and C.

**FIGURE 12:** Job position and O.

In addition, the author also conducted a simple test on the variation trend between Education level/Age and HEXACO. After that, two conclusions could be got. Firstly, there is generally a positive correlation between education level and H-H/X/C/O. Meanwhile, there is a general negative correlation between Education level and E/A. That is to say that, when there is an upward trend in the education level, H-H/X/C/O is likely to have a corresponding strengthening momentum, and E/A may correspondingly have a weakened momentum. Secondly, age and H-H/X/C/O have a general positive correlation. Simultaneously, there is a general negative correlation between Age and E/A. It means that when there is an upward trend in age, H-H/X/C/O is likely to have a corresponding strengthening momentum, and E/A may correspondingly have a weakened momentum.

The five main variables covered in the offline interview questionnaire can all be examined visually through the Shapiro–Wilk test and visualization. That is to say, all valid data collected about offline interviews can pass the normality test. Therefore, the hypothesis proposed in this study can be verified by the bivariate correlation analysis. Table 4 reflects the correlation of employees’ personality traits measured by HEXACO and their annual salaries. By carefully observing the results of the correlation analysis reflected in Table 4, it is easy to find the following conclusions:

**TABLE 4:** The bivariate correlation of employees’ personality traits and their annual salary.

Variables	Annual salary	H-H	E	X	A	C	O
Annual salary	1.000	0.966***	−0.972***	0.968***	−0.974***	0.965***	0.971***
H-H	0.966***	1.000	–	–	–	–	–
E	−0.972***	–	1.000	–	–	–	–
X	0.968***	–	–	1.000	–	–	–
A	−0.974***	–	–	–	1.000	–	–
C	0.965***	–	–	–	–	1.000	–
O	0.971***	–	–	–	–	–	1.000

***Indicates that the correlation coefficient passes the significance test of the 0.01 level. –Indicates null value. H-H, E, X, A, C, and O represent a personality trait in HEXACO, respectively.

Firstly, H-H has a positive association with employees’ annual salaries significantly.

Secondly, E has a negative association with employees’ annual salaries significantly.

Thirdly, X has a positive association with employees’ annual salaries significantly.

Fourthly, A has a negative association with employees’ annual salaries significantly.

Fifthly, C has a positive association with employees’ annual salaries significantly.

Finally, O has a positive association with employees’ annual salaries significantly.

Thus, employees’ annual salaries co-increase with the strengthening of H-H, X, C, and O (referring to an increase in numerical values). Meanwhile, employees’ annual salaries could rise with the weakening of E and A (referring to a decline in numerical values). In other words, H-H, X, C, and O all have a positive co-movement with employees’ annual salaries significantly. So H1, H3, H5, and H6 could be accepted and verified. At the same time, E and A have a negative co-movement with employees’ annual salaries significantly which means that H2 and H4 could pass the test and be accepted.

## Conclusion

Personality traits have a non-negligible impact on personal economic status (De Haro et al., 2020). In order to further reveal the quantitative relationship between the two, researchers investigated individuals’ personality traits and the income of some specific subjects through questionnaires (Kräft and Urgelles, 2021). Subsequently, they used quantitative analysis to verify the correlation between personality traits and personal incomes (Nyhus and Pons, 2005). From the perspective of the scale they used, the previous quantitative studies on personal financial outcomes preferred using the Big Five scale to investigate the personality traits of specific research groups (Judge et al., 1999; Kräft and Urgelles, 2021). Compared with HEXACO, the Big Five has a significant defect in measuring personality traits (Ludeke et al., 2019). It lacks a critical dimension called H-H, which HEXACO listed. From the perspective of the objects, most previous quantitative research focused on the active employees of general companies or college graduates who have just entered the workplace (Kräft and Urgelles, 2021). Compared with these two groups, it seems that the leading group of this study (active employees in Chinese startups) is more concrete and targeted.

Based on these, this research designed two questionnaires (an online questionnaire and an offline interview questionnaire) to investigate the employees’ annual income (before tax), education level, position, age, and personality traits measured by HEXACO in detail. Then, with the assistance of correlation and regression analysis, the quantitative relationship among personality traits, personal education level, individual job position, and private annual salary (before tax) was explored. Through the results, it is easy to find the following conclusion. The six personality traits in HEXACO all significantly correlated with an individual’s annual salary. In detail, H-H, X, C, and O positively correlated with personal annual salary, while E and A negatively correlated with it.

Judging from the present results, in Chinese startups, the more significant the H-H, X, C, and O of an active employee, the more annual salary he or she may obtain. Conversely, the more remarkable the E and A of an active employee, the less annual salary he or she may get. Therefore, for an active employee (worked for Chinese startups) who wants to increase their annual salaries by transferring their personality, deliberately sharping their competitiveness in H-H, X, C, and O, and weakening their features in E and A purposely, might be an effective approach.

It is worth mentioning that this paper is the first to verify the correlation between H-H and personal annual salary, finding that the former positively correlates with the latter significantly. So, it not only makes up for the shortcomings of previous studies in H-H but also lays a specific foundation for using the HEXACO scale to research the quantitative relationship between personality traits and personal income.

Overall, this study has three limitations. Firstly, the sample size is relatively small. Due to the limited time and energy of the author, only 376 valid sample data were collected. Secondly, the survey mainly focuses on employees of Chinese startups and does not involve other countries. Therefore, the conclusions drawn in this paper have limited applicability in the international context. Thirdly, the participants in this survey may conceal their true thoughts to a certain extent while filling out the questionnaire and accepting offline interviews due to “social expectations” or other causes. Moreover, the companies surveyed in this paper mainly concentrate on Jiangsu province and Zhejiang province (South of China). Considering that there are noticeable regional differences in Chinese economic and cultural development between the South and North, the results of this study may not be applied to interpreting the current employees of all startups in China.

Given the above limitations, future research can be developed in the following aspects: Firstly, further expanding the sample size. Secondly, researching the relationship between personality characteristics and the annual income of employees of startups in different regions of China and verifying whether the conclusions of this paper are still applicable in other provinces of China. Thirdly, taking startups in other countries (except China) as examples and exploring the correlation between employees’ personalities and annual salaries.

## Data availability statement

The raw data supporting the conclusions of this article will be made available by the authors, without undue reservation.

## Ethics statement

Ethical review and approval was not required for the study on human participants in accordance with the local legislation and institutional requirements. Written informed consent from the patients/participants or patients/participants legal guardian/next of kin was not required to participate in this study in accordance with the national legislation and the institutional requirements.

## Author contributions

The author confirms being the sole contributor of this work and has approved it for publication.
